This article has been retracted.

# A Hyperglycemic Microenvironment Inhibits Tendon-to-Bone Healing through the let-7b-5p/CFTR Pathway

**DOI:** 10.1155/2022/8268067

**Published:** 2022-01-27

**Authors:** Tianyi Cao, Junyi Hong, Feicheng Qi, Bo Zheng, Guofang Chen, Binjia Yu, Fusheng Ye

**Affiliations:** Department of Orthopedics, Affiliated Xiaoshan Hospital, Hangzhou Normal University, China

## Abstract

**Background:**

Tendon-to-bone healing is a difficult process in treatment of rotator cuff tear (RCT). In addition, diabetes is an important risk factor for poor tendon-to-bone healing. Therefore, we investigated the specific mechanisms through which diabetes affects tendon-to-bone healing by regulating the Cystic Fibrosis Transmembrane Conductance Regulator (CFTR).

**Methods:**

Tendon-derived stem cells (TDSCs) were extracted from rats after which their proliferative capacities were evaluated by the MTT assay. The expression levels of CFTR and tendon-related markers were determined by qRT-PCR. Then, bioinformatics analyses and dual luciferase reporter gene assays were used to identify miRNAs with the ability to bind CFTR mRNA. Finally, CFTR was overexpressed in TDSCs to validate the specific mechanisms through which the high glucose microenvironment inhibits tendon-to-bone healing.

**Results:**

The high glucose microenvironment downregulated mRNA expression levels of tendon-related markers and CFTR in TDSCs cultured with different glucose concentrations. Additionally, bioinformatics analyses revealed that let-7b-5p may be regulated by the high glucose microenvironment and can regulate CFTR levels. Moreover, a dual luciferase reporter gene assay was used to confirm that let-7b-5p targets and binds CFTR mRNA. Additional experiments also confirmed that overexpressed CFTR effectively reversed the negative effects of the hyperglycaemic microenvironment and upregulation of let-7b-5p on TDSC proliferation and differentiation. These findings imply that the hyperglycemic microenvironment inhibits CFTR transcription and, consequently, proliferation and differentiation of TDSCs *in vitro* by upregulating let-7b-5p.

**Conclusions:**

A hyperglycemic microenvironment inhibits TDSC proliferation *in vitro* via the let-7b-5p/CFTR pathway, and this is a potential mechanism in diabetes-induced poor tendon-to-bone healing.

## 1. Introduction

The rotator cuff tear (RCT), a common disorder of the locomotor system, causes shoulder pain and dysfunction [1]. Notably, tendon-to-bone healing is a difficult aspect in RCT treatment, with approximately 11-36% of patients experiencing as a disease that affects hundreds of millions of people [2, 3]. This disease is a significant risk factor for tendinopathy. In addition, approximately 40% of diabetic patients are less likely to recover from tendon-related injuries [4]. Moreover, many musculoskeletal disorders, such as RCT, are likely to occur in diabetics than in nondiabetics [4–8]. Diabetic patients are at a higher risk of tendon-to-bone injury due to structural changes in the tendon, caused by the hyperglycemic microenvironment [5, 9]. Hyperglycemia is also a risk factor for rotator cuff tears [10]. Diabetic patients have also been associated with poor prognostic outcomes with regard to postoperative tendon injury and are less able to heal [11, 12]. However, the exact mechanisms through which diabetes induces poor tendon-to-bone healing remain unclear.

Tendon-derived stem cells (TDSCs) have been identified in various mammalian tendon tissues. They exhibit stem cell properties, including a multidirectional differentiation potential, self-renewal ability, and clonogenicity [13]. TDSCs play a key role in tendon homeostasis and have been shown to promote the regeneration and repair of tendon injuries [14, 15]. Among other factors, the correct differentiation and proliferation of TDSCs is key in tendon-to-bone healing [16, 17]. The current development of tissue engineering is generating increasingly promising applications for the treatment of motor system disorders [18–20]. Additionally, TDSCs have been shown to overcome the disadvantages of ectopic ossification of bone marrow mesenchymal stem cells and have been considered as the most ideal seed cells for tendon tissue engineering [21–23]. The hyperglycemic microenvironment in diabetics inhibits the healing of diabetic tendon injuries by affecting TDSC proliferation and differentiation [10, 24]. Therefore, investigation of specific mechanisms through which the hyperglycemic microenvironment affects TDSCs may be beneficial in improvising ways to improve tendon-to-bone healing in diabetic patients.

The Cystic Fibrosis Transmembrane Conductance Regulator (CFTR) acts as a chloride channel, controlling the movement of chloride ions or water into and out of cells [25]. Therefore, dysfunction in CFTR affects normal intercellular signaling pathways and is associated with the progression of various diseases. CFTR has potential mechanosensitive gating properties [26]. Therefore, mechanical stimulation has been shown to promote tendon differentiation through gene expressions and protein synthesis in TDSCs [27, 28]. Moreover, CFTR is associated with various diseases of the locomotor system (e.g., myasthenia gravis, reduced bone density, and cartilage abnormalities). Interestingly, recent studies report that CFTR promotes TDSC proliferation and proper differentiation [29], confirming its importance in tendon-to-bone healing. Studies have confirmed the role of CFTR in diabetes [30], and its downregulation is associated with insulin deficiency and overactivation of the body's inflammatory responses [31]. Therefore, we hypothesized that the hyperglycemic microenvironment plays a role in poor tendon-to-bone healing in diabetic patients by downregulating CFTR-mediated impairments of TDSC proliferation and differentiation.

MiRNAs are endogenous single-stranded RNAs with the ability to regulate gene expressions by binding specific sequences of target mRNAs. Additionally, posttranscriptional expression of CFTR is regulated by miRNAs [32, 33]. For instance, Bartoszewska et al. showed that miR-200b was able to downregulate the expression of CFTR in lung epithelial cells [34]. MicroRNAs are also involved in regulation of insulin and blood glucose levels during diabetes pathogenesis and are closely associated with fat metabolism as well as the development of obesity [35]. Diabetes is also involved in regulating the damage from motor system disorders through miRNAs [35, 36]. Therefore, the hyperglycemic microenvironment may affect CFTR transcription, thereby downregulating TDSC proliferation and differentiation by regulating miRNA expressions. This may be a potential mechanism for treating diabetes-induced poor tendon-to-bone healing.

In this study, we investigated the specific mechanisms through which diabetes affects tendon-to-bone healing by regulating the Cystic Fibrosis Transmembrane Conductance Regulator (CFTR). Additionally, we investigated the specific mechanisms involved in diabetes-miRNA-CFTR regulation at the cellular level. This was done to identify the potential targets for improving poor tendon-to-bone healing in diabetic patients.

## 2. Materials and Methods

### 2.1. Experimental Animals

Thirty-six 7-8 weeks old Sprague-Dawley rats (purchased from Shanghai Super, B&K Laboratory Animal Corp. Ltd.) were used in this study. Animals were housed in a light/dark (12 h/12 h) cycle, controlled temperature (22–25°C) environment, with free access to water and food. The food was replaced every 2-3 days to prevent spoiling. Ambient humidity was 55 ± 5%. Animal refusal to physical activity was used as a preexclusion criterion. None of the animals were excluded or euthanized before completing the experiments. To reduce animal suffering, their welfare, experimental procedures, and criteria for euthanasia were performed in strict accordance with Guidelines for the Management and Use of Laboratory Animals (Chinese Ministry of Science and Technology, 2006). Under normal physiological conditions, animals with dying or sickness symptoms were euthanized. At the end of the experiment, all animals were euthanized with Thiopental sodium (150 mg/kg). This study was approved by the Animal Research Ethics Committee.

### 2.2. Isolation and Culture of Rat TDSCs

TDSCs were isolated from rat patellar tendon tissues as previously described [13, 24]. Briefly, rats were anesthetized with an overdose of 2.5% phenobarbital. Thereafter, tissues from the midpatellar tendon were excised, and connective tissues surrounding the sample carefully removed. On the first day, the tissue was minced and digested with collagenase type I (3 mg/mL; Sigma-Aldrich) after which a single cell suspension was obtained using a 70 *μ*m cell filter (Becton Dickinson, Franklin Lakes, NJ). Then, cells were washed using sterile phosphate-buffered saline (PBS) at 37°C in a constant environment of 5% CO_2_ then seeded in a medium (10% fetal bovine serum, 100 U/mL penicillin, 100 mg/mL streptomycin, Dulbecco's Modified Eagle Medium (DMEM, low glucose formulation. Glucose concentration: 5.5 mM)) (Invitrogen Corporation, Carlsbad, CA) at an optimally low cell density. On the second day, cells were washed using PBS to remove nonadherent cells, and on day seven, they were trypsinized and mixed. Moreover, cell status was confirmed using previously described assays. The medium was changed every 3 days [13]. In this experiment, the DMEM medium with different glucose concentrations was used to investigate the effects of different glucose concentrations on TDSCs. The obtained cells were equally randomized into 12 groups according to the experimental design. Randomization was performed by the double-blind principle.

### 2.3. Lentivirus Transfection

A lentiviral system was successfully constructed as described previously [37]. Briefly, the coding region of CFTR was cloned downstream of the promoter of the pCDH plasmid in cytomegalovirus. In addition, CHIP or control lentiviral plasmids were cotransfected into HEK293T cells after which lentiviral supernatants were collected 48 h after transfection. Then, TDSCs were transfected with the lentivirus in the presence of 6 *μ*g/mL polyethylene (Sigma, St. Louis, USA).

### 2.4. Transfection of miRNAs

Transfection of miRNAs was performed according to a previously published protocol [38]. Chemically synthesized let-7b-5p mimics and let-7b-5p inhibitors (Gene Pharma (Shanghai, China)) were used to enhance and inhibit the biological functions of let-7b-5p. Then, cells were inoculated and transfected for 24 h using the riboFECT™ CP transfection kit, according to the manufacturer's instructions (Ribobio, Guangzhou, China). Thereafter, real-time fluorescence quantitative PCR was performed after 48 h to ascertain the efficiency of transfection.

### 2.5. Luciferase Reporter Assay

First, let-7b-5p mimics or inhibitors (GenePharma) and HEK293T cells were first cotransfected with the recombinant plasmid in triplicates. In addition, cells were lysed after 24 h of transient transfection using Lipofectamine 2000 (Invitrogen), according to the manufacturer's instructions. Moreover, firefly and Renilla luciferase activities were measured using the Dual-Luciferase Reporter Assay System (Promega).

### 2.6. Quantitative Real-Time RT-PCR

Total RNA was isolated from samples (using the RNeasy Plus Mini kit (Qiagen)) after which the superscript first strand synthesis SuperMix kit (Invitrogen) was used for reverse transcription to obtain cDNA. Thereafter, real-time fluorescent quantitative RT-PCR analysis was performed using SYBR Green. In addition, miRNA isolation was performed using TRIzol® reagents (Gibco/Life 270 Technologies, Thermo Fisher Scientific) followed by detection of miRNA quantity and quality (detected using the stem-loop quantitative RT-PCR (TaqMan probe method)). Purified miRNA was used for first-strand cDNA synthesis using the M-MLV reverse transcriptase and primers, according to the manufacturer's instructions (Promega, Fitchberg, MA, USA). The primer sequences were as follows: CFTR forward: 5′-AAGTCGAGTCCAACCTGAACC-3′, backward 5′-TTGGTGTGGTCCAGCTGAAGA-3′; Internal reference *β*-actin forward 5′-CCGTGAAAAGATGACCC-3′, backward 5′-AGAGGCATACAGGGACAACA-3′; U6, forward: 5′-GCTTCGG CAGCACATATACT-3′, backward: 5′-GTGCAGGGTCCGAGGTATTC-3.

### 2.7. Western Blotting

Total proteins were isolated from cultured cells using a RIPA lysis buffer (Thermo Fisher Scientific) and a 1% protease inhibitor (Roche). Proteins were separated by SDS-PAGE and transferred to PVDF membranes using the semidry method. Thereafter, the membrane was blocked using 5% fat-free milk for 1 h and incubated overnight with primary antibodies at 4°C. The primary antibodies were anti-CFTR (1 : 1000, ab181782; ABCAM), B-catenin resistance (1 : 1000, 610053; BD Biosciences), anti-phosphoric acid-B-catenin (1 : 500, YP-0047; Immunoway, Plano, TX, USA), and anti-GAPDH (1 : 10000, SC-25778; Santa Cruz Biotechnology). Then, the membrane was washed in Tris-buffered saline containing Tween 20 after which it was incubated with horseradish peroxidase–conjugated secondary antibodies (anti-mouse or anti-rabbit; Santa Cruz Biotechnology) for 1 h at room temperature. The blot was developed using the Amersham ECL Western Blotting Detection Reagent (GE Healthcare, Waukesha, WI, USA), according to the manufacturer's instructions [29].

### 2.8. MTT Assays

Cell survival and proliferation rates were determined using the MTT assay. Briefly, TDSCs were seeded at a density of 3 × 10^3^ cells/well in 96-well culture plates for 24 h. After aspiration of the complete medium, cells were cultured in complete medium containing different glucose concentrations (25 mM, 15 mM, and 5.5 mM). Thereafter, the MTT assays were performed on days 1, 3, and 5. The MTT assays were performed as follows: DMEM containing 5 mg/mL of MTT (Sigma-Aldrich, USA) was added into each well and incubated at 37°C for 4 h. The MTT solution was removed before adding 150 *μ*L of dimethyl sulfoxide (DMSO (Sigma-Aldrich, USA)) into each well. Following this, crystals were dissolved by mixing using a micropipette after which absorbance at 570 nm was measured using 150 *μ*L of DMSO (Sigma-Aldrich, USA), immediately after the DMSO turned purple [29]. All experiments were performed in triplicates.

### 2.9. Enrichment Analysis of Genes Targeted by let-7c-5p

The miRTarBase database is a dedicated collection of microRNA-mRNA targeting relationships (MTI, MicroRNA-Target Interactions) supported by experimental evidence. The database was used to predict potential target genes for let-7c-5p [39, 40]. GO and KEGG enrichment analysis was done using the clusterProfiler package (version 3.14.3) [41, 42]. The http://org.Hs.eg.db package (version 3.10.0) was used for ID conversion; the GOplot package (version 1.0.2) was used to calculate the zscore. The top ranked pathways were filtered out and visualised and analysed using the R software.

### 2.10. Bioinformatics and Statistical Analysis

Data on the potentially relevant CFTR miRNAs was obtained from the GSE114828 dataset in the GEO database (http://www.ncbi.nlm.nih.gov/geo/) and raw data from a previous study [43]. It is noteworthy that the GSE114828 dataset is the only miRNA microarray of TDSCs that documents miRNAs that are potentially associated with tendinopathy [44]. In addition, Ying et al. fully investigated diabetes-associated microRNAs, and it was from their study that the raw data herein were obtained [43]. Therefore, we used the two studies to obtain miRNAs that were jointly associated with tendinopathy and diabetes. Moreover, correlations between CFTR and miRNAs were assessed using the miRWalk3.0 database (http://mirwalk.umm.uni-heidelberg.de/), which includes 10 databases (Targetscan, RNA22, PITA, PICTAR5, PICTAR4, RNAhybrid, miRWalk, miRDB, miRanda, and DIANAmT). Additionally, GSEA is a database (http://www.bio-info-trainee.com/3705.html) for investigating potential mechanisms using JAVA (http://software.broadinstitute.org/gsea/index.jsp) [45]. Besides, the GTEX database contains gene expression signatures in normal human samples and is used for GSEA analysis as well as investigation of coexpression signatures, to investigate the functional characteristics of genes. Furthermore, the sample random parameter was set at 500, and *p* ≤ 0.05 was considered to be statistically significant.

Data are expressed as mean ± standard deviation. Statistical analyses and graphing were performed using GraphPad Prism (version 7.0). Comparisons of statistical differences among and between groups were performed by one-way ANOVA and two-tailed *t*-tests, respectively. *p* ≤ 0.05 was considered to be statistically significant.

## 3. Results

### 3.1. Hyperglycemia Inhibited Cell Proliferation and Suppressed the Expressions of Key Tendon-Related Markers of TDSCs

TDSCs were cultured in medium with different glucose concentrations after which their activities were measured by the MTT assay (Figure 1(a)). There was a significant decrease in the proliferative rate of cells after treatment with a high concentration of glucose. Differences in proliferative cells between the normal group (glucose concentration 5.5 mM) and the high glucose concentration group (glucose concentration 15 mM or 25 mM) were significant. Moreover, qRT-PCR assays showed that expressions of CFTR, Tnmd, Col-l, and Scx mRNAs were significantly downregulated in the groups treated with 15 mM and 25 mM of glucose, relative to the normoglycemic category (Figure 1(b)). These results indicate that the high glucose microenvironment downregulated the mRNA expressions of tendon-related markers and CFTR in TDSCs. Furthermore, expressions of the CFTR protein were downregulated in the high glucose environment (15 mM and 25 mM; Figures 1(c) and 1(d)).

### 3.2. Let-7b-5p Targets and Regulates CFTR in a Hyperglycemic Microenvironment

To the best of our knowledge, currently, the GSE114828 dataset is the only miRNA dataset that documents the lesions associated with TDSCs. Intersections of CFTR-related miRNAs, T2DM-related miRNAs, and TDSCs-related miRNAs were shown by the VEEN plot (Figure 2(a)). Let-7b-5p levels were downregulated in normal TDSCs, relative to diseased TDSCs (Figure 2(b)). In contrast, let-7b-5p was upregulated in diabetic patients (Figure 2(c)). Let-7b-5p was also downregulated in TDSCs treated with 15 mM and 25 mM of glucose (Figure 2(d)). This suggested that let-7b-5p may target and regulate CFTR in hyperglycemic microenvironments. The RNA hybrid 2.12 was used to predict the binding site of let-7b-5p and CFTR at the 3′UTR (Figure 2(e)) while a dual luciferase reporter gene assay was used to confirm that let-7b-5p targeted and bound the CFTR mRNA. Luciferase activities of TDSCs transfected with wild-type CFTR and let-7b-5p mimics were significantly low than those of TDSCs transfected with mutant CFTR and let-7b-5p mimics (Figure 2(f)). In contrast, the let-7b-5p inhibitor upregulated the expressions of CFTR (Figure 2(g)). Therefore, it is possible that let-7b-5p targets and regulates CFTR in a hyperglycemic microenvironment.

### 3.3. Enrichment Analysis of let-7b-5p Target Genes

To further determine the potential biological function of let-7b-5p, we used the miRTarBase database to identify currently known target genes for let-7b-5p. A total of 1204 target genes for let-7b-5p were identified. These genes were used for further enrichment analysis (Figure 3). GO enrichment analysis identified Biological Processes (BPs) that were significantly enriched for let-7c-5p target genes including positive regulation of catabolic process, response to acid chemical, and response to ionizing radiation. Cellular Component (CC) was significantly enriched for serine/threonine protein kinase complex, cyclin-dependent protein kinase holoenzyme complex, and protein kinase complex. The significantly enriched Molecular Function (MF) includes mRNA 5′-UTR binding, cyclin-dependent protein serine/threonine kinase regulator activity, and histone binding. In addition, pathways of neurodegeneration-multiple diseases, p53 signaling pathway, and FoxO signaling pathway were found to be the main enrichment KEGG pathways for let-7c-5p target gene enrichment.

### 3.4. A Hyperglycemic Microenvironment Downregulates CFTR by Upregulating let-7b-5p

TDSCs were cultured in a high glucose (25 mM) medium after which associations between cell activities and let-7b-5p were evaluated by the MTT assay (Figure 4(a)). The let-7b-5p inhibitor significantly upregulated the proliferative capacities of TDSCs in a high glucose environment, while the let-7b-5p mimic significantly downregulated the proliferative capacities of TDSCs. In addition, overexpressed CFTR upregulated the proliferative capacities of TDSCs and reversed the inhibition of TDSCs-activities that were as a result of the hyperglycemic microenvironment and the let-7b-5p mimic (Figure 4(b)). These findings imply that let-7b-5p affects the activities of TSDCs by influencing CFTR expressions. Moreover, Western blot showed that upregulated CFTR protein levels, caused by overexpression of CFTR, were suppressed by the let-7b-5p mimic and DMEM (high glucose), as shown in Figure 4(c). The qRT-PCR assays also showed that overexpressed CFTR was able to upregulate the expressions of CFTR, Tnmd, and Col-l mRNAs. Expressions of CFTR, Tnmd, Col-l, and Scx mRNAs were upregulated by overexpressions of CFTR while upregulations of CFTR, Tnmd, Col-l, and Scx mRNAs were suppressed by the let-7b-5p mimic and DMEM (high glucose), as shown in Figure 4(d). Therefore, the hyperglycemic microenvironment downregulated CFTR by upregulating let-7b-5p.

## 4. Discussion

We used an *in vitro* high-glucose microenvironment model to show, for the first time, that a high-glucose microenvironment upregulates the expressions of let-7b-5p and CFTR. These findings imply that CFTR is an upstream regulatory protein of markers related to tendon formation (Tnmd, Col-l, and Scx). In addition, CFTR transcription was directly regulated by let-7b-5p while its overexpression effectively reversed the negative regulatory effects caused by the hyperglycemic microenvironment and upregulation of let-7b-5p on TDSC proliferation and differentiation. In summary, a hyperglycemic microenvironment inhibits CFTR transcription *in vitro* by upregulating let-7b-5p and may play a role in suppressing TDSC proliferation and differentiation.

The specific mechanisms through which diabetes leads to poor tendon-to-bone healing remain highly unclear. However, TDSCs have been shown to be potential key model cells for studying tendon-to-bone healing mechanisms [21, 22]. In addition, expressions of key biomarkers for tendon differentiation, including Tnmd, Col-l, and Scx, are important indicators for TDSC differentiation [29, 37, 46]. Elevated Scx and Tnmd levels, which are key molecules in tendon development, are prerequisites for the differentiation and formation of tendon cells [47]. In this study, the hyperglycemic microenvironment was able to inhibit the expressions of key biomarkers of tendon differentiation, consistent with previous studies [24].

CFTR promotes TDSC proliferation and differentiation [29], implying its importance in tendon-to-bone healing. We established that the hyperglycemic microenvironment downregulated the expressions of CFTR and tendon-related markers (Tnmd, Col-l, and Scx) in TDSCs. In contrast, overexpressed CFTR upregulated the expressions of tendon-related markers (Tnmd, Col-l, and Scx). In previous studies, pathogenic mechanisms of CFTR abnormalities in hyperglycaemic microenvironments and downregulations of CFTR were associated with insulin deficiency as well as overactivated inflammatory responses [30, 31]. We found that the ability to inhibit the proliferation and differentiation of TDSCs by the hyperglycaemic microenvironment may be dependent on downregulation of CFTR expression.

miRNAs are important mediators of cell differentiation and act as key regulators of disease development and pathological processes [48, 49]. In this study, let-7b-5p was found to be downregulated in diseased TDSCs but upregulated in diabetic patients. The dual luciferase reporter gene assays confirmed that let-7b-5p targets and binds the CFTR mRNA. Additionally, Western blot assays showed that let-7b-5p mimics downregulate CFTR protein levels in TDSCs. Therefore, it is possible that let-7b-5p targets and regulates CFTR in hyperglycemic microenvironments. Let-7b-5p is associated with diabetic cardiomyopathy and mitochondrial damage [50, 51]. In addition, let-7b-5p inhibits the growth and development of skeletal muscles while its downregulation promotes the accumulation vitamin D, thereby preventing muscle damage [52, 53]. In this study, effects of let-7b-5p/CFTR on TDSC differentiation and proliferation were investigated. The MTT assay confirmed that let-7b-5p was negatively correlated with cell proliferation as well as activities and inhibited the expressions of Tnmd, Col-l, and Scx, the key biomarkers for myotendinous differentiations. However, overexpressions of CFTR effectively reversed the negative effects of high glucose microenvironments and upregulations of let-7b-5p on TDSC proliferation and differentiation.

In summary, we used *in vitro* experiments and bioinformatics analyses to explore regulatory relationships between hyperglycemic microenvironments, let-7b-5p, CFTR, and TDSCs. Therefore, future studies should use animal models to validate if hyperglycemic microenvironments regulate TDSC proliferation and differentiation via the let-7b-5p/CFTR pathway. In addition, clinical studies should be performed to screen and validate diabetic-induced tendon-to-bone malhealing. In the future, single cell technology may be used for further studies of the tendon to bone healing process due to its spatial and temporal specificity [8, 54–56]. Transcriptional regulation regarding CFTR and let-7c should also be used for further studies in the future [57–60].

## 5. Conclusions

Hyperglycemic microenvironments inhibit TDSC proliferation *in vitro* via the let-7b-5p/CFTR pathway and suppress the expressions of tendon-related markers. Therefore, for the first time, we show the potential mechanisms and therapeutic targets for diabetes-induced poor tendon-to-bone healing.

## Figures and Tables

**Figure 1:** Hyperglycemia inhibited cell proliferation and suppressed the expression of key tendon-related markers of TDSCs. (a) TDSCs were cultured in different glucose concentrations (5.5 mM, 15 mM, and 25 mM), and cell activities were measured by the MTT assay. (b) qRT-PCR assays showed that expressions of CFTR, Tnmd, Col-l, and Scx mRNAs were significantly downregulated in 15 mM and 25 mM glucose-treated cells, relative to the normoglycemic group (*p* < 0.05). (c) A high glucose microenvironment downregulated the mRNA expressions of tendon-related markers and CFTR in TDSCs. (d) Expressions of the CFTR protein were downregulated in the high glucose environment (15 mM and 25 mM).

**Figure 2:** Let-7b-5p targets and regulates CFTR in a hyperglycemic microenvironment. (a) Intersections of CFTR-related miRNAs, T2DM-related miRNAs, and TDSCs-related miRNAs were shown by the VEEN plot. (b) A volcanic map of miRNAs related to TDSCs. (c) Relative expression levels of let-7b-5p in the diabetic and normal groups. (d) Expressions of let-7b-5p were significantly upregulated after high glucose (15 mM and 25 mM) treatment of TDSCs, compared to the control (5.5 mM), *p* < 0.05. (e). Let-7b-5p targeting regulated CFTR transcription, as predicted by RNAhybrid (minimum free energy = −28.9 kcal/mol). (f). TDSCs were transfected with the 3′UTR CFTR luciferase reporter gene along with a let-7b-5p mimic or let-7b-5p inhibitor, respectively. (g) Western blot assays demonstrated that the let-7b-5p mimic significantly downregulated CFTR protein levels in TDSCs.

**Figure 3:** Histogram of Let-7c-5p target gene enrichment analysis.

**Figure 4:** A hyperglycemic microenvironment downregulated CFTR by upregulating let-7b-5p. (a). TDSCs were cultured in a high glucose (25 mM) medium after which cell activities in relation to let-7b-5p were evaluated by the MTT assay. (b) Treatment of TDSCs with DMEM (high glucose), overexpressed CFTR and the let-7b-5p mimic, reduced cell proliferations on days 1, 3, and 5. (c) Western blot analysis showed that upregulations of CFTR protein expressions, caused by overexpressed CFTR, were suppressed by the let-7b-5p mimic and DMEM (high glucose). (d) qRT-PCR assay showed that overexpressed CFTR upregulated CFTR, Tnmd, Col-l, and Scx mRNA levels. In addition, the let-7b-5p mimic and DMEM (high glucose) suppressed the upregulation of CFTR, Tnmd, Col-l, and Scx, caused by the overexpressed CFTR; ^∗^*p* < 0.05.

## Data Availability

Original data from this study can be obtained by contacting the corresponding author.

## Abbreviations

CFTR: Cystic Fibrosis Transmembrane Conductance Regulator
DE-miRNAs: Differentially expressed microRNAs
EV: Empty vector
GEO: The Gene Expression Omnibus
NC: Normal control
TDSCs: Tendon-derived stem cells
T2DM: Type 2 diabetes mellitus.

## References

[1] Mather R. C., Koenig L., Acevedo D. (2013). The societal and economic value of rotator cuff repair. *The Journal of Bone and Joint Surgery. American Volume*.

[2] Galatz L. M., Griggs S., Cameron B. D., Iannotti J. P. (2001). Prospective longitudinal analysis of postoperative shoulder function: a ten-year follow-up study of full-thickness rotator cuff tears. *The Journal of Bone and Joint Surgery. American Volume*.

[3] Zandi H., Coghlan J. A., Bell S. N. (2006). Mini-incision rotator cuff repair: a longitudinal assessment with no deterioration of result up to nine years. *Journal of Shoulder and Elbow Surgery*.

[4] Ranger T. A., Wong A. M., Cook J. L., Gaida J. E. (2016). Is there an association between tendinopathy and diabetes mellitus? A systematic review with meta-analysis. *British Journal of Sports Medicine*.

[5] Bedi A., Fox A. J., Harris P. E. (2010). Diabetes mellitus impairs tendon-bone healing after rotator cuff repair. *Journal of Shoulder and Elbow Surgery*.

[6] Kalyanaraman H., Schwaerzer G., Ramdani G. (2018). Protein kinase G activation reverses oxidative stress and restores osteoblast function and bone formation in male mice with type 1 diabetes. *Diabetes*.

[7] Marin C., Luyten F. P., Van der Schueren B., Kerckhofs G., Vandamme K. (2018). The impact of type 2 diabetes on bone fracture healing. *Frontiers in Endocrinology*.

[8] Chen Y. S., Cai Y. X., Kang X. R. (2020). Predicting the risk of sarcopenia in elderly patients with patellar fracture: development and assessment of a new predictive nomogram. *Peer J*.

[9] Fox A. J., Bedi A., Deng X. H. (2011). Diabetes mellitus alters the mechanical properties of the native tendon in an experimental rat model. *Journal of Orthopaedic Research*.

[10] Shi L., Rui Y. F., Li G., Wang C. (2015). Alterations of tendons in diabetes mellitus: what are the current findings?. *International Orthopaedics*.

[11] Maffulli N., Longo U. G., Maffulli G. D., Khanna A., Denaro V. (2011). Achilles tendon ruptures in diabetic patients. *Archives of Orthopaedic and Trauma Surgery*.

[12] Brophy R. H., Wright R. W., Huston L. J., Nwosu S. K., Spindler K. P. (2015). Factors associated with infection following anterior cruciate ligament reconstruction. *The Journal of Bone and Joint Surgery. American Volume*.

[13] Rui Y. F., Lui P. P., Li G., Fu S. C., Lee Y. W., Chan K. M. (2010). Isolation and characterization of multipotent rat tendon-derived stem cells. *Tissue Engineering. Part A*.

[14] Chen Y., Sun Y., Xu Y. (2021). Single-cell integration analysis of heterotopic ossification and fibrocartilage developmental lineage: endoplasmic reticulum stress effector Xbp1 transcriptionally regulates the notch signaling pathway to mediate fibrocartilage differentiation. *Oxidative Medicine and Cellular Longevity*.

[15] Lui P. P., Wong O. T., Lee Y. W. (2016). Transplantation of tendon-derived stem cells pre-treated with connective tissue growth factor and ascorbic acid in vitro promoted better tendon repair in a patellar tendon window injury rat model. *Cytotherapy*.

[16] Ni M., Lui P. P., Rui Y. F. (2012). Tendon-derived stem cells (TDSCs) promote tendon repair in a rat patellar tendon window defect model. *Journal of Orthopaedic Research*.

[17] Zhang X., Lin Y. C., Rui Y. F. (2016). Therapeutic roles of tendon stem/progenitor cells in tendinopathy. *Stem Cells International*.

[18] Han Z., Wang Q., Wu X. (2021). Comprehensive RNA expression profile of therapeutic adipose-derived mesenchymal stem cells co-cultured with degenerative nucleus pulposus cells. *Molecular Medicine Reports*.

[19] Leppik L., Sielatycka K., Henrich D. (2020). Role of adult tissue-derived pluripotent stem cells in bone regeneration. *Stem Cell Reviews and Reports*.

[20] Ying J., Han Z., Pei S., Su L., Ruan D. (2019). Effects of stromal cell-derived factor-1*α* secreted in degenerative intervertebral disc on activation and recruitment of nucleus pulposus-derived stem cells. *Stem Cells International*.

[21] Chen J., Zhang W., Liu Z. (2016). Characterization and comparison of post-natal rat Achilles tendon-derived stem cells at different development stages. *Scientific Reports*.

[22] Leone L., Raffa S., Vetrano M. (2016). Extracorporeal shock wave treatment (ESWT) enhances the in vitro-induced differentiation of human tendon-derived stem/progenitor cells (hTSPCs). *Oncotarget*.

[23] Dressler M. R., Butler D. L., Boivin G. P. (2005). Effects of age on the repair ability of mesenchymal stem cells in rabbit tendon. *Journal of Orthopaedic Research*.

[24] Lin Y. C., Li Y. J., Rui Y. F. (2017). The effects of high glucose on tendon-derived stem cells: implications of the pathogenesis of diabetic tendon disorders. *Oncotarget*.

[25] Cutting G. R. (2015). Cystic fibrosis genetics: from molecular understanding to clinical application. *Nature Reviews. Genetics*.

[26] Zhang W. K., Wang D., Duan Y., Loy M. M., Chan H. C., Huang P. (2010). Mechanosensitive gating of CFTR. *Nature Cell Biology*.

[27] Nourissat G., Berenbaum F., Duprez D. (2015). Tendon injury: from biology to tendon repair. *Nature Reviews Rheumatology*.

[28] Ni M., Rui Y. F., Tan Q. (2013). Engineered scaffold-free tendon tissue produced by tendon-derived stem cells. *Biomaterials*.

[29] Liu Y., Xu J., Xu L. (2017). Cystic fibrosis transmembrane conductance regulator mediates tenogenic differentiation of tendon-derived stem cells and tendon repair: accelerating tendon injury healing by intervening in its downstream signaling. *The FASEB Journal*.

[30] Norris A. W. (2019). Is cystic fibrosis-related diabetes reversible? New data on CFTR potentiation and insulin secretion. *American Journal of Respiratory and Critical Care Medicine*.

[31] Hart N. J., Aramandla R., Poffenberger G. (2018). Cystic fibrosis-related diabetes is caused by islet loss and inflammation. *Insight*.

[32] Gillen A. E., Gosalia N., Leir S. H., Harris A. (2011). MicroRNA regulation of expression of the cystic fibrosis transmembrane conductance regulator gene. *The Biochemical Journal*.

[33] De Palma F. D. E., Raia V., Kroemer G., Maiuri M. C. (2020). The multifaceted roles of microRNAs in cystic fibrosis. *Diagnostics*.

[34] Bartoszewska S., Kamysz W., Jakiela B. (2017). miR-200b downregulates CFTR during hypoxia in human lung epithelial cells. *Cellular & Molecular Biology Letters*.

[35] Improta Caria A. C., Nonaka C. K. V., Pereira C. S., Soares M. B. P., Macambira S. G., Souza B. S. F. (2018). Exercise training-induced changes in microRNAs: beneficial regulatory effects in hypertension, type 2 diabetes, and obesity. *International Journal of Molecular Sciences*.

[36] Chen Y. S., Kang X. R., Zhou Z. H. (2020). MiR-1908/EXO1 and MiR-203a/FOS, regulated by scd1, are associated with fracture risk and bone health in postmenopausal diabetic women. *Aging*.

[37] Han W., Chen L., Liu J., Guo A. (2017). Enhanced tenogenic differentiation and tendon-like tissue formation by CHIP overexpression in tendon-derived stem cells. *Acta Biochim Biophys Sin (Shanghai)*.

[38] Zhou Z., Lu Y., Wang Y., Du L., Zhang Y., Tao J. (2019). Let-7c regulates proliferation and osteodifferentiation of human adipose-derived mesenchymal stem cells under oxidative stress by targeting SCD-1. *American Journal of Physiology. Cell Physiology*.

[39] Chou C. H., Shrestha S., Yang C. D. (2018). miRTarBase update 2018: a resource for experimentally validated microRNA-target interactions. *Nucleic Acids Research*.

[40] Hsu S. D., Lin F. M., Wu W. Y. (2011). miRTarBase: a database curates experimentally validated microRNA-target interactions. *Nucleic Acids Research*.

[41] Yu G., Wang L. G., Han Y., He Q. Y. (2012). clusterProfiler: an R package for comparing biological themes among gene clusters. *OMICS*.

[42] Walter W., Sánchez-Cabo F., Ricote M. (2015). GOplot: an R package for visually combining expression data with functional analysis. *Bioinformatics*.

[43] Liang Y. Z., Dong J., Zhang J., Wang S., He Y., Yan Y. X. (2018). Identification of neuroendocrine stress response-related circulating microRNAs as biomarkers for type 2 diabetes mellitus and insulin resistance. *Frontiers in Endocrinology*.

[44] Geng Y., Zhao X., Xu J. (2020). Overexpression of mechanical sensitive miR-337-3p alleviates ectopic ossification in rat tendinopathy model via targeting IRS1 and Nox4 of tendon-derived stem cells. *Journal of Molecular Cell Biology*.

[45] Subramanian A., Tamayo P., Mootha V. K. (2005). Gene set enrichment analysis: a knowledge-based approach for interpreting genome-wide expression profiles. *Proceedings of the National Academy of Sciences of the United States of America*.

[46] Dunkman A. A., Buckley M. R., Mienaltowski M. J. (2014). The tendon injury response is influenced by decorin and biglycan. *Annals of Biomedical Engineering*.

[47] Jiang Y., Shi Y., He J. (2017). Enhanced tenogenic differentiation and tendon-like tissue formation by tenomodulin overexpression in murine mesenchymal stem cells. *Journal of Tissue Engineering and Regenerative Medicine*.

[48] Bartoszewska S., Kochan K., Madanecki P. (2013). Regulation of the unfolded protein response by microRNAs. *Cellular & Molecular Biology Letters*.

[49] Wang Y., Zhao Z. J., Kang X. R. (2020). lncRNA DLEU2 acts as a miR-181a sponge to regulate SEPP1 and inhibit skeletal muscle differentiation and regeneration. *Aging*.

[50] Li H., Dai B., Fan J. (2019). The different roles of miRNA-92a-2-5p and let-7b-5p in mitochondrial translation in db/db mice. *Mol Ther Nucleic Acids*.

[51] Marques F. Z., Vizi D., Khammy O., Mariani J. A., Kaye D. M. (2016). The transcardiac gradient of cardio-microRNAs in the failing heart. *European Journal of Heart Failure*.

[52] Araujo H. N., Lima T. I., Guimarães D. (2020). Regulation of Lin28a-miRNA let-7b-5p pathway in skeletal muscle cells by peroxisome proliferator-activated receptor delta. *American Journal of Physiology. Cell Physiology*.

[53] Yu H. M., Yao X. D., Zhang R. M., Zhuang H. F., Wang P. W., Li Y. Z. (2019). Repression of let-7b-5p prevents the development of multifidus muscle dysfunction by promoting vitamin D accumulation via upregulation of electron transfer flavoprotein alpha subunit in a rat model of multifidus muscle injury. *Journal of Cellular Biochemistry*.

[54] De Micheli A. J., Swanson J. B., Disser N. P. (2020). Single-cell transcriptomic analysis identifies extensive heterogeneity in the cellular composition of mouse Achilles tendons. *American Journal of Physiology. Cell Physiology*.

[55] Kang X., Chen Y., Yi B. (2021). An integrative microenvironment approach for laryngeal carcinoma: the role of immune/methylation/autophagy signatures on disease clinical prognosis and single-cell genotypes. *Journal of Cancer*.

[56] Wu J. Y., Qin J., Li L. (2021). Roles of the immune/methylation/autophagy landscape on single-cell genotypes and stroke risk in breast cancer microenvironment. *Oxidative Medicine and Cellular Longevity*.

[57] Xinbing L., Wei G., Wei L. (2021). Identification of KLF6/PSGs and NPY-related USF2/CEACAM transcriptional regulatory networks via spinal cord bulk and single-cell RNA-Seq analysis. *Disease Markers*.

[58] Aibar S., González-Blas C. B., Moerman T. (2017). SCENIC: single-cell regulatory network inference and clustering. *Nature Methods*.

[59] Lin W. W., Xu L. T., Chen Y. S., Go K., Sun C., Zhu Y. J. (2021). Single-cell transcriptomics-based study of transcriptional regulatory features in the mouse brain vasculature. *BioMed Research International*.

[60] Zhang P., Liu B. (2021). Integrative bioinformatics analysis reveals that infarct-mediated overexpression of potential miR-662/CREB1 pathway-induced neuropeptide VIP is associated with the risk of atrial fibrillation: a correlation analysis between myocardial electrophysiology and neuroendocrine. *Disease Markers*.

